This article has been retracted.

# Application of Deep Neural Network Factor Analysis Model in Operating Room Management Nursing Analysis of Postoperative Infection Nursing after Thoracic Surgery

**DOI:** 10.1155/2021/4622064

**Published:** 2021-10-26

**Authors:** Jing Wen, Jun He

**Affiliations:** ^1^Department of Medical Engineering, Tangshan Workers' Hospital, Hebei Province, China 063000; ^2^Department of Thoracic Surgery, Tangshan Workers' Hospital, Hebei Province, China 063000

## Abstract

Thoracic surgery is the main surgical method for the treatment of respiratory diseases and lung diseases, but infections caused by improper care are prone to occur during the operation, which can induce pulmonary edema and lung injury and affect the effect of the operation and the subsequent recovery. Therefore, it is necessary to control the disease in time and adopt more scientific and comprehensive nursing measures. Based on the neural network algorithm, this paper constructs a neural network-based factor analysis model and applies the operating room management nursing to postoperative infection nursing after thoracic surgery and verifies the effect through the neural network model. The statistical parameters in this article mainly include the postoperative infection rate of thoracic surgery, patient satisfaction, postoperative rehabilitation effect, and complications. Through statistical analysis, it can be known that operating room management and nursing can play an important role in postoperative infection nursing after thoracic surgery, effectively reducing postoperative infection nursing after thoracic surgery, and improving the recovery effect of patients after infection.

## 1. Introduction

Nosocomial infection (NI) is also known as hospital-acquired infection. It refers to infections acquired by hospitalized patients in the hospital, including infections that occurred during hospitalization and infections acquired in the hospital after discharge, but does not include infections that have begun before admission or existed at the time of admission. Nowadays, with the development of medical science; the advancement of medical technology; the development of radiotherapy and chemotherapy for malignant tumor diseases; the popularization and application of invasive treatment; the widespread and universal use of immunosuppressants, cytotoxic drugs, and antibacterial drugs; and the morbidity and mortality of the disease itself have been significantly reduced, but nosocomial infections have always existed [1].

Thoracic surgery can disrupt the central nervous system of the body due to the long operation time, large trauma of the patient, and residual anesthetic drugs in the operation, resulting in postoperative discomfort for the patient. Moreover, patients have varying degrees of restlessness and confusion, and severe cases may lead to various accidental injuries, such as incision dehiscence, various catheters falling off, and bed falling, which affect the patient's smooth recovery from general anesthesia [2]. Second, the postoperative infection will not only impair the operation's effectiveness, lengthen the patient's stay in the hospital, and raise treatment expenses, but it will also pose a risk to the patient's life in extreme instances [3].

In the hospital quality management system, the operating room quality management is one of the important management systems. All types of surgery, treatment, and emergency rescue of surgical patients are carried out in the operating room, so the operating room is more demanding than the quality management of the outpatient and inpatient areas. Furthermore, since the operating theatre entails a high level of risk and complexity, its quality management is linked not only to the lives of surgical patients but also to the quality of surgical output services [4].

At present, China has taken various preventive measures to prevent the occurrence of nosocomial infections and established a nationwide nosocomial infection monitoring system to monitor the status of nosocomial infections, effectively reducing the incidence of nosocomial infections. However, adverse events caused by hospital infections still occur from time to time.

Regarding the monitoring and control of nosocomial infections, we can use different methods to measure the intensity of nosocomial infections. There are also many risk factors that cause nosocomial infections, such as the research objects used for comparison and reference, the control of confounding factors, and the difference in the length of hospital stay [5]. As a result, effective confounding factor control and differentiation, accurate measurement of nosocomial infection incidence, timely identification of hospitalized patients at high risk of infection, and analysis of risk factors for nosocomial infections can determine the key direction of nosocomial infection surveillance and control and effectively reduce the incidence of nosocomial infections. At present, domestic research on nosocomial infection of patients undergoing thoracic surgery is relatively scattered, and most of them are small sample studies and retrospective investigations. Moreover, single-factor analysis is adopted for nosocomial infection risk factors, and multifactor research is few, and the research results are relatively scattered.

This paper constructs a factor analysis model based on neural network algorithm and applies operating room management nursing to postoperative infection nursing after thoracic surgery. Furthermore, this paper uses a neural network model to verify the impact, and it serves as a reference for postoperative infection nursing in thoracic surgery.

## 2. Related Work

Nosocomial infection monitoring refers to long-term, systematic and continuous observation, collection and analysis of the occurrence, and distribution of nosocomial infections in a certain population and its influencing factors, and the monitoring results are reported and fed back to relevant units and individuals. Moreover, it is the basis and basis for the prevention and control measures of nosocomial infection. Nosocomial infection monitoring can provide data to assess the size of the problem, determine the risk factors of nosocomial infection, provide effective control methods for high-risk patients, or evaluate the effects of preventive measures [5]. The ultimate aim is to decrease the number of nosocomial infections while still ensuring patient safety. Nosocomial infection monitoring may be split into two types: comprehensive monitoring and focused monitoring, depending on the monitoring goals and scope.

Comprehensive monitoring is to monitor the nosocomial infections and related influencing factors of all inpatients and staff in the whole hospital from many aspects to understand the occurrence of nosocomial infections in the whole hospital, which requires a lot of time and human resources. As early as 1970, at the first international infection conference held in the United States, the importance of nosocomial infection surveillance was raised by people. After formulating the infection control plan, the United States took the lead in establishing the world's first nosocomial infection surveillance system, the National Nosocomial Infection Surveillance (NNIS). By 2000, 315 hospitals had joined the NNIS.

Various nations' nosocomial infection surveillance systems conduct surveillance with different foci based on the epidemiological features of nosocomial illnesses in their respective countries. However, the majority of them, such as the NNIS system, can explain the epidemiology of nosocomial infections, antibacterial drug resistance, quantify the frequency of nosocomial infections, and conduct hospital comparisons [6].

Nosocomial infections in thoracic surgery are mainly the respiratory tract, accounting for about 64.82% [7]. There are more patients with tumors in thoracic surgery and elderly patients, and most of them are accompanied by respiratory diseases. The respiratory function itself is damaged to a certain degree, and it is prone to coughing weakness, difficulty in expectoration, and sputum retention, which are all causes of respiratory infections. Among patients with nosocomial infections, the highest hospitalization costs are patients with lower respiratory tract infections, with an average hospitalization cost of 24,693 yuan, and the longest average hospital stay of patients with hospital infections is also lower respiratory tract infection, with an average stay of 22.2 days [8].

According to the findings of the literature [9], urinary system infections are the most common hospital infections in Europe and the United States, followed by infections of the surgical site, skin and mucous membranes, and the lower respiratory tract. The results of nosocomial infection survey of patients undergoing thoracic surgery showed that the constituent ratio of urinary tract infection was 1.32%-22.32%, and the average length of stay for urinary tract infection was the shortest at 7.7 days [10].

Surgery site infection (SSI) is one of the most common complications after surgery. Thoracic surgery has large surgical wounds and more invasive procedures, and most of the illnesses are critically ill, and the probability of SSI is high. SSI refers to infections that occur in the deep organs or cavities of the incision or surgery during the perioperative period. It includes ① superficial surgical incision infection: it is limited to the skin and subcutaneous tissue involved in the incision, and the infection occurs within 30 days after surgery. ② For infection of deep surgical incision, it occurs 30 days after surgery without implants and within 1 year after surgery with implants (such as artificial heart valves, artificial blood vessels, mechanical hearts, and artificial joints). It is a surgical infection that affects the incision's deep soft tissues (deep fascia and muscle). ③ For organ (or cavity) infection, it occurs 30 days after surgery without implants and within 1 year after surgery with implants (such as artificial heart valves, artificial blood vessels, mechanical hearts, and artificial joints). It is an infection of organs or cavities related to surgery (except skin, subcutaneous, deep fascia, and muscle) [11].

Isolation of pathogenic bacteria based on pathogenic specimens submitted by hospital-infected patients can understand the distribution and trend of pathogenic bacteria causing hospital infections and help doctors choose antibacterial drugs reasonably. At present, most of the pathogens causing nosocomial infections in thoracic surgery patients are Gram-negative bacilli, followed by Gram-positive cocci and fungi. The distribution composition ratio of pathogenic bacteria varies slightly with the investigation hospital. Among them, the main ones are Pseudomonas aeruginosa, Staphylococcus aureus, and Candida albicans [12].

Malnutrition is often linked with cancer patients. All components of the immune system may be harmed when a patient is malnourished, and the intensity of the effect is generally equal to the severity of the malnutrition. When patients are malnourished, nosocomial infections are common [13]. This is due to malnutrition leading to low immunity and susceptibility to conditional pathogens, which can cause hospital infections [14]. The surgical site infection rate of malnourished patients is 22.41%, which is much higher than that of ordinary patients [15].

The rate of nosocomial infection caused by diabetes and the mortality rate of nosocomial infection are very high, respectively, 20.63% and 1.68% [16]. Zhao Yuehua's research showed that the postoperative nosocomial infection rate of general surgery patients with diabetes is 18.72%, which is much higher than that of patients without diabetes (5.92%) during the same period. Moreover, postoperative nosocomial infections are mainly caused by surgical incision infections, followed by respiratory infections. In a study of infection at the surgical site, it was also shown that excellent blood glucose management before surgery may decrease infection problems in a variety of surgical operations [17]. In addition, glycosylated hemoglobin (HbAlc) can be used as one of the monitoring indicators of high-risk factors for nosocomial infection in diabetic patients, and its stability is better than fasting blood glucose [18–20].

## 3. RBM Related Variant Algorithms

RBM is generally only suitable for processing binary data. Therefore, many scholars later proposed a series of RBM variant algorithms to process real-valued data, such as Gaussian RBM (GRBM), covariance RBM (cRBM), mean and covariance RBM (mcRBM), and spike and flat RBM (ssRBM).

GRBM is the earliest proposed RBM variant model for modeling real-valued data. It regards the visible layer unit of traditional RBM as a Gaussian variable with diagonal covariance. In this way, the energy function of GRBM is redefined as:

(1) $$\begin{array}{c} E\left(v,h;\theta \right)=-\overset{D}{\underset{i=1}{\sum }}\overset{J}{\underset{j=1}{\sum }}\frac{v_{i}}{\sigma_{i}}W_{ij}h_{j}-\overset{J}{\underset{j=1}{\sum }}b_{j}h_{j}+\overset{D}{\underset{i=1}{\sum }}\frac{{\left(v_{i}-c_{i}\right)}^{2}}{2\sigma_{i}^{2}}. \end{array}$$

Among them, *σ*_*i*_^2^ represents the variance term on the *i*-th visible layer unit. Then, when any one of the visible and hidden layers in GRBM is in a fixed state, the conditional probability distribution of the other layer can be calculated:

(2) $$\begin{array}{c} P\left(v_{i}\left|h\right.\right)=\frac{1}{\sigma_{i}\sqrt{2\pi }}\cdot \exp\left(-\frac{1}{2\sigma_{i}^{2}}\left(v_{i}-c_{i}-\sigma_{i}\underset{j}{\sum }W_{ij}h_{j}\right)\right), \end{array}$$

(3) $$\begin{array}{c} P\left(h_{j}=1\left|v\right.\right)=\sigma \left(\underset{i}{\sum }\frac{v_{i}}{\sigma_{i}}W_{ij}+b_{j}\right). \end{array}$$

Among them,

(4) $$\begin{array}{c} \sigma \left(x\right)=\frac{1}{\left(1+\exp\left(-x\right)\right)}, \end{array}$$

represents the sigmoid activation function. In this way, *P*(*v*_*i*_|*h*) can be expressed in terms of *N*(*σ*_*i*_∑_*j*_*W*_*ij*_*h*_*j*_ + *c*_*i*_, *σ*_*i*_^2^); that is, it conforms to a Gaussian distribution with mean *σ*_*i*_∑_*j*_*W*_*ij*_*h*_*j*_ + *c*_*i*_ and variance *σ*_*i*_^2^. In this way, when GRBM uses the CD algorithm to train the network model, the gradient of the parameter {*W*, *b*, *c*, *σ*} can be expressed as:

(5) $$\begin{array}{c} \Delta W_{ij}=\frac{\alpha \left(\sum_{n=1}^{N}\left(v_{i}^{n}/\sigma_{i}\right)h_{j}^{n0}-\sum_{n=1}^{N}\left(v_{i}^{n}/\sigma_{i}\right)h_{j}^{nk}\right)}{N}, \end{array}$$

(6) $$\begin{array}{c} \Delta b_{j}=\frac{\alpha \left(\sum_{n=1}^{N}h_{j}^{n0}-\sum_{n=1}^{N}h_{j}^{nk}\right)}{N}, \end{array}$$

(7) $$\begin{array}{c} \Delta c_{i}=\frac{\alpha \left(\sum_{n=1}^{N}\left(v_{i}^{n}/\sigma_{i}^{2}\right)-\sum_{n=1}^{N}\left(v_{i}^{nk}/\sigma_{i}^{2}\right)\right)}{N}, \end{array}$$

(8) $$\begin{array}{c} \Delta \sigma_{i}=\frac{\alpha_{\sigma }}{N}\left(\begin{array}{c} \overset{N}{\underset{n=1}{\sum }}\left(\frac{{\left(v_{i}^{n}-c_{i}\right)}^{2}}{\sigma_{i}^{3}}-\overset{J}{\underset{j=1}{\sum }}\frac{v_{i}^{n}W_{ij}h_{j}^{n}}{\sigma_{i}^{2}}\right)-\\ \overset{N}{\underset{n=1}{\sum }}\left(\frac{{\left(v_{i}^{nk}-c_{i}\right)}^{2}}{\sigma_{i}^{3}}-\overset{J}{\underset{j=1}{\sum }}\frac{v_{i}^{n}W_{ij}h_{j}^{nk}}{\sigma_{i}^{2}}\right) \end{array}\right). \end{array}$$

ssRBM is a variant of RBM based on GRBM and cRBM for modeling real-valued data. It uses two types of hidden layers to determine the mean and covariance of each visible unit, and it can also use block Gibbs sampling to calculate the state of the visible unit. In this way, the energy function of ssRBM is redefined as:

(9) $$\begin{array}{c} E\left(v,s,h;\theta \right)=\frac{1}{2}v^{T}\Lambda v-\overset{j}{\underset{j=1}{\sum }}\left(v^{T}W_{j}s_{j}h_{j}+\frac{1}{2}s_{j}\alpha_{j}s_{j}+b_{j}h_{j}\right). \end{array}$$

Among them, *W*_*j*_ represents the column vector of the *j*-th column of the matrix *W*, and *α* and *Λ* are diagonal matrices, which are used to punish the larger values in the ‖*s*‖_2_^2^ and ‖*v*‖_2_^2^ terms, respectively. Then, the conditional probability distribution in ssRBM can be expressed as:

(10) $$\begin{array}{c} P\left(h_{j}=1\left|v\right.\right)=\sigma \left(\frac{1}{2}v^{T}W_{j}\alpha_{j}W_{j}^{T}+b_{j}\right), \end{array}$$

(11) $$\begin{array}{c} P\left(s_{j}\left|v,h\right.\right)\sim N\left(h_{j}\alpha_{j}^{-1}W_{j}^{T}v,\alpha_{j}^{-1}\right), \end{array}$$

(12) $$\begin{array}{c} P\left(v\left|s,h,\left\|v\right\|\leq R\right.\right)\sim N\left(\Lambda^{-1}\overset{j}{\underset{j=1}{\sum }}W_{j}s_{j}h_{j},\Lambda^{-1}\right). \end{array}$$

Among them, *N*(*μ*, *σ*^2^) represents a Gaussian distribution with mean *μ* and variance *σ*^2^, and ‖*v*‖ ≤ *R* in *P*(*v*|*s*, *h*, ‖*v*‖ ≤ *R*) represents rejection of sampling when ‖*v*‖ is too large.

RBM is a generative model, and data generation also helps to denoise data, such as Point-wise Gated RBM (pgRBM) and Robust GRBM (Robust GRBM, RoGRBM). As shown in Figure 1, pgRBM and RoGRBM adjust the network model and energy function of RBM to better achieve image denoising and recognition tasks. The noisy picture that pgRBM can analyze is one with background noise that cannot obscure the portion of the image that is relevant to classification. RoRBM, on the other hand, can learn the structure of noise in noisy pictures using noise-free photos to accomplish image denoising.

The pgRBM network has three levels: a visible layer, a conversion layer, and two hidden layers, as illustrated in Figure 1(a). pgRBM splits the hidden layer nodes into two categories: classification-related and classification-unrelated. It can identify the classification-related portions of the data in the background data in an adaptive manner. Simultaneously, it uses unsupervised learning to extract hidden layer features in this portion of the data, resulting in improved classification results. In this way, the energy function of pgRBM is defined as:

(13) $$\begin{array}{c} \begin{array}{c} E\left(v,z,h^{1},h^{2};\theta \right)=-\overset{D}{\underset{i=1}{\sum }}\overset{J}{\underset{j=1}{\sum }}\overset{2}{\underset{r=1}{\sum }}\left(z_{i}^{r}v_{i}\right)W_{ij}^{r}h_{j}^{r}-\\ \overset{J}{\underset{j=1}{\sum }}\overset{2}{\underset{r=1}{\sum }}b_{j}^{r}h_{j}^{r}-\overset{D}{\underset{i=1}{\sum }}\overset{2}{\underset{r=1}{\sum }}c_{i}^{r}\left(z_{i}^{r}v_{i}\right)\\ \text{s}.\text{t}.\overset{2}{\underset{r=1}{\sum }}z_{i}^{r}=1.i=1,\vdots ,D. \end{array} \end{array}$$

Among them, *h*^1^ represents a hidden layer related to classification, and *h*^2^ represents a hidden layer not related to classification. Then, the conditional probability distribution in pgRBM can be expressed as:

(14) $$\begin{array}{c} P\left(h_{j}^{r}=1\left|z,v\right.\right)=\sigma \left(\underset{i}{\sum }\left(z_{i}^{r}v_{i}\right)W_{ij}^{r}+b_{j}^{r}\right), \end{array}$$

(15) $$\begin{array}{c} P\left(v_{i}=1\left|z,h^{1},h^{2}\right.\right)=\sigma \left(\underset{r}{\sum }z_{i}^{r}\left(\underset{j}{\sum }W_{ij}^{r}h_{j}^{r}+c_{i}^{r}\right)\right), \end{array}$$

(16) $$\begin{array}{c} P\left(z_{i}^{r}=1\left|v,h^{1},h^{2}\right.\right)=\frac{\exp\left(v_{i}\left(\sum_{j}W_{ij}^{r}h_{j}^{r}+c_{i}^{r}\right)\right)}{\sum_{s}\exp\left(v_{i}\left(\sum_{j}W_{ij}^{s}h_{j}^{s}+c_{i}^{s}\right)\right)}. \end{array}$$

Unlike traditional RBM, the initial value of pgRBM is not randomly generated. After the network weights obtained by RBM learning (the number of hidden layer nodes in RBM is slightly larger than the sum of the number of hidden layer nodes in pgRBM), it then uses the feature selection method to determine the contribution of the hidden layer nodes to the classification based on the label of the sample to determine the initial value of the pgRBM network weight.

## 4. Research Methods

The study selected 124 patients undergoing thoracic surgery in the undergraduate room as the subjects of this survey. The selected time for the survey was from January 2019 to December 2020. The patients participating in the survey were divided into two groups by lottery, the control group and the test group, and the number of patients in each group was 62. In the control group, there are 30 males and 32 males, and they are 33-65 years old, with an average of 49.6 ± 4.5 years old. There are 29 male and 33 male patients in the test group, and the age ranged from 33 to 66 years old, with an average of 49.2 ± 4.5 years old. Moreover, all patients had 28 cases of education below junior high school, accounting for 35.90%. There is no statistically significant difference in general information between the control group and the test group (*P* > 0.05), and all patients must have thoracic surgery following diagnosis. All members of the ethics committee gave their approval to this inquiry. Both patients and their families were aware of this survey and volunteer to participate. Inclusion criteria are the following: patients who take part in the survey are aware of it and consent to it, they are all patients who need thoracic surgery, and they do not have any cognitive or mental disorders. Criteria for exclusion are the following: patients or family members are aware of the survey but refuse to take part because they have cognitive or mental disorders. The control group was given routine nursing operations.

Before the surgery, the patients were examined, the operation plan was explained to them in detail, venous access was created for them, the physicians were helped in the operation throughout the procedure, and the patients were given routine care such as medicine after the operation. The test group gave patients interventional care in the operating room: (1) Before the operation, the nursing staff should strengthen the understanding of the patient's specific information, and according to the understanding of the patient, ensure that the patient has a good mood and actively cooperate with the treatment. The specific nursing method is to understand the basic information of the patient in detail, conduct a comprehensive analysis of the patient's condition, and explain in detail the problems and precautions that may be encountered during the operation, so that the patient has a scientific and comprehensive understanding of the disease. Furthermore, medical personnel aggressively encourage patients and inform them about successful instances in order to instil faith in the disease's cure and urge patients to actively participate in therapy. At the same time, it is necessary to ensure that the operating room environment is quiet and tidy, and the temperature is appropriate to keep the patient nervous. (2) After entering the room, the nursing staff should inform the operation procedure and strengthen communication with the patient at the same time. The particular nursing technique is to expose the patient to the operating room atmosphere, massage the patient's limbs, and say something calming to the patient to alleviate the patient's stress. At the same time, it is necessary to pay attention to the patient's expression during the whole process and deal with it in time. During the operation, it is necessary to strictly carry out the correct operation and sterility awareness, pay close attention to the changes in the patient's vital signs and mental state, and find and deal with the accidents that occur during the operation as soon as possible. (3) After the operation, the relevant nursing staff strengthened the prevention and control of lung infection. The specific nursing measures are to closely monitor the patient's vital signs and lung function to prevent abnormal conditions. Moreover, it is necessary to actively guide the patient's diet, etc., and instruct the patient's diet to gradually transition from water to liquid food and then to a normal diet. In addition, nurses need to help patients knock their backs on time, instruct patients to breathe properly, keep patients' airways unobstructed, inform patients that smoking is strictly prohibited, and ask patients' families to pay attention to patients' emotional state, keep warm, and actively encourage patients.

The control group's patients were all given standard treatment initially. At the same time, it is essential to pay attention to the signs and keep track of them, educate patients about key things to remember before and after the surgery, help the doctor in finishing the procedure, and securely transport the patient to the ward. Forty patients in the test group were given high-quality nursing care in the operating room on the basis of routine nursing. The main nursing measures are as follows. First of all, preoperative high-quality nursing patients will be evaluated in their psychological and physical aspects after admission to learn more about the patient's medical history and provide targeted care plans. If the patient has a history of smoking, it is necessary to introduce the hazards of smoking and cooperate with the doctor to instruct them to quit smoking. Simultaneously, patients must be encouraged, their reasons of illness and treatment methods explained, typical instances of successful surgery shown, and their faith in the operation's success boosted. The patient's transfer procedure must be gentle, with little turbulence, and keep the patient warm in order to provide high-quality intraoperative care. If necessary, a scarf can be placed around the patient's neck, and the patient's quilt can be removed when the doctor is preparing for disinfection. In addition, it is necessary to provide patients with a high-quality environment during the operation as much as possible. The laminar flow unit is turned on half an hour before the operation to purify the air in the operating room, and various disinfection tasks are strictly carried out. In high-quality postoperative care, the patient needs to be in a semirecumbent position after anesthesia is sober and blood pressure stabilizes. Moreover, it is necessary to help patients turn over and pat their backs every 2 hours, encourage and help patients cough and expectorate, and instruct patients to protect their hands when coughing to relieve pain. At the same time, it is necessary to help patients perform deep breathing exercises to ensure unobstructed airway, increase lung capacity, promote lung expansion, improve lung function, and closely monitor patients for lung infections. In addition, it is necessary to pay attention to whether the patient has new coughs, the frequency of coughs, and changes in the nature of sputum.

## 5. Results

This article analyzes the application of operating room management in postoperative infection care after thoracic surgery through the above test analysis and combines the deep neural network analysis model to perform data processing. The statistical parameters in this article mainly include the postoperative infection rate of thoracic surgery, patient satisfaction, postoperative rehabilitation effect, and complications. The research results are statistically studied.

The test group's and control group's postoperative infection rates were calculated, and the results are presented in Table 1 and Figure 2. Among them, 1 means infection, and 0 means no infection.

The use of operating room management nursing in postthoracic surgery infection nursing may successfully decrease the postthoracic surgery infection rate, according to the statistical analysis of the above trials. Afterwards, the postoperative patient satisfaction of the test group and the control group was counted. The results obtained are shown in Table 2 and Figure 3.

From the statistical analysis of the above experiments, we can see that the application of operating room management nursing in postoperative infection nursing after thoracic surgery can effectively improve patient satisfaction. After that, the rehabilitation effects of postoperative patients in the test group and the control group were calculated. The results obtained are shown in Table 3 and Figure 4.

The use of operating room management nursing in postoperative infection nursing after thoracic surgery may significantly enhance the postoperative rehabilitation impact, according to the statistical analysis of the above trials. Afterwards, the postoperative complications of the test group and the control group were counted. The results obtained are shown in Table 4 and Figure 5; 1 means that complications occurred, and 0 means that no complications occurred.

From the statistical analysis of the above experiments, it can be seen that the application of operating room management nursing in postoperative infection nursing after thoracic surgery can effectively reduce the occurrence of postoperative complications in patients.

In summary, operating room management and nursing can play an important role in postoperative infection nursing after thoracic surgery.

## 6. Conclusion

The number of patients admitted to the operating room has shown an upward trend year by year. From an environmental point of view, the operating room is a special place where surgical treatment is concentrated, and it is more prone to cross-infection compared with conventional wards. Among them, surgical wound infection is a relatively common complication in surgical patients. Wound infection will directly affect the patient's treatment time and bring certain effects to the patient. Effective clinical nursing for patients during surgery can promote the prognosis of patients, increase the recovery speed of patients, and reduce the occurrence of postoperative complications. Moreover, the application of human-centered nursing and comfort nursing in operating room nursing can improve the overall nursing effect. Comfort care is primarily concerned with providing nursing services to patients based on their current circumstances and reducing the development of problems via excellent psychological and physical nursing. In addition, in the nursing process, it is necessary to adhere to the people-oriented approach, try to meet the needs of patients, and improve the quality of nursing.

## Figures and Tables

**Figure 1:** Network structure of (a) pgRBM and (b) RoGRBM algorithm models.

**Figure 2:** Statistical diagram of postoperative infection rate after thoracic surgery.

**Figure 3:** Statistical diagram of patient satisfaction after thoracic surgery.

**Figure 4:** Statistical diagram of rehabilitation effect of patients after thoracic surgery.

**Figure 5:** Statistical diagram of complications of patients after thoracic surgery.

**Table 1:** Statistical table of postoperative infection rate after thoracic surgery.

No.	Control group	Test group	No.	Control group	Test group
1	0	0	32	0	0
2	0	0	33	0	0
3	1	0	34	1	0
4	0	1	35	0	0
5	0	0	36	0	0
6	0	0	37	0	1
7	0	1	38	0	0
8	0	0	39	0	0
9	1	0	40	0	0
10	0	0	41	0	0
11	0	0	42	0	0
12	0	0	43	0	0
13	0	0	44	0	0
14	0	0	45	0	0
15	0	0	46	0	0
16	1	0	47	0	0
17	0	0	48	1	0
18	0	0	49	0	0
19	0	0	50	0	0
20	1	0	51	0	0
21	0	0	52	0	0
22	1	1	53	0	0
23	0	0	54	1	0
24	0	0	55	0	0
25	0	0	56	0	0
26	1	0	57	0	0
27	0	0	58	0	0
28	0	0	59	0	0
29	0	0	60	0	0
30	0	0	61	0	0
31	0	0	62	1	1

**Table 2:** Statistical table of patient satisfaction after thoracic surgery.

No.	Control group	Test group	No.	Control group	Test group
1	91	87	32	0	0
2	83	93	33	0	0
3	87	84	34	1	0
4	92	83	35	0	0
5	87	84	36	0	0
6	83	93	37	0	1
7	84	90	38	0	0
8	91	83	39	0	0
9	87	89	40	0	0
10	92	96	41	0	0
11	82	95	42	0	0
12	85	86	43	0	0
13	90	84	44	0	0
14	91	85	45	0	0
15	83	94	46	0	0
16	83	88	47	0	0
17	84	98	48	1	0
18	76	98	49	0	0
19	87	87	50	0	0
20	85	87	51	0	0
21	81	88	52	0	0
22	77	86	53	0	0
23	80	92	54	1	0
24	86	98	55	0	0
25	89	86	56	0	0
26	78	89	57	0	0
27	84	96	58	0	0
28	88	89	59	0	0
29	78	89	60	0	0
30	74	90	61	0	0
31	79	84	62	1	1

**Table 3:** Statistical table of rehabilitation effect of patients after thoracic surgery.

No.	Control group	Test group	No.	Control group	Test group
1	93.9	95.3	32	91.1	96.8
2	94.9	93.2	33	94.7	84.9
3	82.6	89.7	34	84.1	98.6
4	91.6	86.1	35	87.0	98.7
5	77.6	89.2	36	81.1	84.1
6	90.4	87.9	37	95.6	89.3
7	76.6	97.2	38	88.0	95.5
8	91.1	96.2	39	96.1	96.9
9	96.6	85.3	40	87.8	90.4
10	87.2	90.0	41	79.9	87.7
11	76.2	86.5	42	87.6	95.0
12	91.7	85.4	43	76.0	92.3
13	94.8	88.9	44	79.7	93.3
14	85.0	95.5	45	87.4	87.2
15	93.4	86.7	46	96.4	92.1
16	89.9	92.7	47	92.4	94.9
17	87.0	96.2	48	86.0	87.9
18	76.6	90.4	49	92.3	90.0
19	96.6	95.9	50	93.0	98.0
20	92.0	95.7	51	84.5	88.1
21	85.3	90.1	52	85.2	96.2
22	88.8	89.8	53	82.2	98.3
23	90.9	88.8	54	95.4	97.2
24	91.3	95.9	55	76.8	85.4
25	82.3	98.1	56	80.0	89.8
26	90.9	86.7	57	94.8	89.5
27	89.0	86.0	58	86.7	91.2
28	94.6	93.9	59	94.4	87.6
29	78.2	89.6	60	83.2	88.5
30	96.5	96.5	61	88.2	95.0
31	79.6	90.7	62	78.1	91.0

**Table 4:** Statistical table of complications of patients after thoracic surgery.

No.	Control group	Test group	No.	Control group	Test group
1	1	1	32	0	0
2	0	0	33	1	0
3	0	0	34	0	0
4	0	0	35	0	0
5	1	0	36	0	0
6	0	0	37	0	0
7	0	0	38	0	0
8	0	0	39	0	0
9	0	0	40	0	0
10	0	0	41	0	0
11	1	0	42	0	0
12	1	0	43	0	0
13	0	0	44	0	0
14	0	0	45	0	0
15	0	0	46	0	0
16	0	1	47	1	0
17	0	0	48	0	0
18	0	0	49	0	0
19	0	0	50	1	0
20	0	0	51	0	0
21	0	0	52	0	0
22	0	0	53	0	0
23	0	0	54	0	1
24	0	0	55	0	0
25	0	0	56	0	0
26	1	0	57	0	0
27	0	0	58	0	0
28	0	0	59	0	0
29	0	1	60	1	0
30	0	0	61	1	1
31	1	0	62	0	0

## Data Availability

The data used to support the findings of this study are included within the article.
